# Computed Tomography Image Feature under Intelligent Algorithms in Diagnosing the Effect of Humanized Nursing on Neuroendocrine Hormones in Patients with Primary Liver Cancer

**DOI:** 10.1155/2021/4563100

**Published:** 2021-10-06

**Authors:** Xiujie Wang, Lin Liu, Na Ma, Xinxin Zhao

**Affiliations:** Department of Gastroenterology, Affiliated Hongqi Hospital of Mudanjiang Medical University, Mudanjiang City 157011, Heilongjiang Province, China

## Abstract

This study was to explore the application value of computed tomography (CT) images processed by intelligent algorithm denoising in the evaluation of humanized nursing in postoperative neuroendocrine hormone changes in patients with primary liver cancer (PLC). In this study, a simple-structured recursive residual coding and decoding (RRCD) algorithm was constructed on the basis of residual network, which can effectively remove artifacts and noise in CT images and can also restore image details and lesion features well. In addition, 60 postoperative patients with primary liver cancer were collected and divided into routine nursing control group (30 cases) and humanized nursing experimental group (30 cases). After a period of nursing, CT images based on intelligent algorithms were evaluated by determining the hormone content. The results showed that the focal necrosis rate (FNR) of the experimental group was 6%. The adrenocorticotropic hormone (ACTH) levels of 6 and 15 days after admission (T3 and T4) were 41.25 ± 3.81 pg/mL and 19.55 ± 1.72 pg/mL, respectively. The cortisol levels of days 6, 15, and 30 after admission (T3, T4, and T5) were 424.86 ± 16.82 nmol/L, 277.98 ± 14.36 nmol/L, and 241.53 ± 13.27 nmol/L, respectively. Estradiol levels were 53.48 ± 11.19 pg/mL, 41.64 ± 9.28 pg/mL, and 30.59 ± 8.16 pg/mL, respectively. Testosterone levels were 2.18 ± 1.14 ng/mL, 1.78 ± 1.03 ng/mL, and 1.42 ± 0.69 ng/mL, respectively. Self-Rating Anxiety Scale (SAS) scores were 40.24 ± 5.81 points, 36.55 ± 5.02 points, and 32.53 ± 4.8 points, respectively. There were 24 cases, 27 cases, 23 cases, and 21 patients who followed no smoking and drinking, taking medication on time, diet control, and self-monitoring. The scores of physical function, self-cognition, emotional function, and social function were 62.59 ± 6.82 points, 69.26 ± 8.14 points, 73.89 ± 6.35 points, and 66.88 ± 7.04 points, which were better than those of the control group in all aspects (*P* < 0.05). In short, the humanized nursing course can enhance the compliance of the patients after the surgery, improve the quality of life, and inhibit the anxiety and depression of the patients, so it showed a positive effect on the neuroendocrine hormones and the prognosis of the patients.

## 1. Introduction

Primary liver cancer (PLC) refers to cancers of liver cells or intrahepatic bile duct cells, which are clinically characterized by persistent pain in the liver area and progressive liver enlargement [1]. PLC is one of the most common malignant tumors in China. The prevalence of PLC is the people aged 40–60 years, and the prevalence of men is higher than that of women. The etiology is usually related to viral hepatitis, liver cirrhosis, aflatoxin, and contaminated drinking water [2]. The main treatment methods include surgery, liquid nitrogen freezing, laser treatment, and so on. However, even if liver cancer is radically removed, 60%–70% of patients still have metastasis and recurrence within 5 years [3], so preventing postoperative recurrence is the key to improving the treatment effect of liver cancer.

In recent years, with the development of psychoneurology, the influence of psychological factors on neuroendocrine has attracted more and more people's attention. Psychological reactions such as anxiety and depression in cancer patients can act as a source of stress, stimulating the body to produce a nonspecific stress response. Based on the neuroendocrine effects, the body's killer cells and T lymphocytes are reduced, thereby causing reduction of immune function in patients with cancer [4, 5]. Many scholars have proposed that the nervousness and anxiety of patients before and after surgery will affect the neuroendocrine and circulatory system, causing a chain reaction such as hyperactivity of sympathetic nerves and increased secretion of catecholamines. In addition, it will cause the immune function of the body to decrease, which will adversely affect the treatment and prognosis of cancer patients [6]. Humanized nursing is a patient-centered nursing concept. Patients with liver cancer have many complications after surgery and are prone to relapse. The patient's physiology and psychology bear a huge burden. Humanized nursing takes care of the physiological and psychological conditions of patients in time and integrates humanistic care into the nursing service, which plays an important role in the recovery of patients after surgery [7, 8].

Computed tomography (CT) is currently a widely used imaging method in the diagnosis of PLC and evaluation of postoperative efficacy. It can display the size, shape, number, blood supply, and extrahepatic metastasis of the liver lesions before and after treatment [9, 10]. However, the accumulation of a large number of X-rays during the examination will increase the probability of illness and cause radiation hazards to the patient. The usual method is to reduce the radiation dose, such as reducing the tube current and incomplete projection, which can greatly reduce the harm of radiation to patients and further expand the scope of application of CT [11, 12]. However, this often causes the final imaging to introduce noise and artifacts, and the quality of CT images is reduced, which affects the diagnosis of the condition by doctors [13]. The residual network is a network structure that can solve the constant performance or even degradation of ordinary convolutional networks when the network is deepened. It regards the noisy image as the aliasing of high-quality image and noise and extracts noise features [14]. In recent years, the residual network has been widely used in CT image denoising. The algorithm can not only save the network training loss but also effectively improve the network performance and reduce the amount of computation during denoising [15], which has good effectiveness and superiority.

In this study, CT imaging technology and hormone content determination method based on intelligent algorithm were applied to 60 patients with PLC after operation. After a period of routine nursing and humanized nursing, the changes of neuroendocrine hormones in patients after operation were comprehensively evaluated, so as to provide reference basis for the treatment and prognosis of PLC and demonstrate the application value of CT imaging in PLC.

## 2. Materials and Methods

### 2.1. Research Objects

A total of 60 PLC patients who underwent surgical treatment at the hospital from February 2019 to March 2021 were selected, and the age range was 35–70 years. They were randomly divided into a conventional nursing control group and humanized nursing experimental group, with 30 cases in each group. The inclusion criteria were defined as follows: patients who complied with the clinical diagnosis and staging criteria of the “PLC Diagnosis and Treatment Specifications” 2017 edition; patients who received the liver cancer surgery for the first time; patients without other serious organic diseases; and patients with complete clinical data.

The exclusion criteria were defined as follows: patients who combined with other malignant tumors; patients with preoperative history of chemotherapy or steroid hormone drugs; women in the menstrual period; patients with incomplete clinical data; patients who did not cooperate with the examination and with poor compliance. This experiment had been approved by the ethics committee of the hospital, and all experimental related matters had been notified to the patient and his family members, and the informed consent forms had been signed.

### 2.2. Nursing Method

Patients in the control group were given postoperative conventional nursing. The patient was informed of postoperative precautions, dietary taboos, and life guidance; it had to pay attention to the patient's consciousness and mental state and be alert for postoperative complications. Patients in the experimental group were given humanized nursing, and the scheme was as follows. (1) *Psychological Nursing.* After the surgery, the nurse should communicate with the patient more, conduct appropriate psychological counseling, listen patiently and respond to the patient's problems, and encourage the patient to relax. In addition, the nurse had to communicate with the patient's family, communicate more with the patient, understand the patient's current inner feelings, and encourage the family to provide more psychological support to the patient. (2) *Drainage Tube Nursing.* A small sticker was adopted as a mark on each drainage tube for easy identification. The nurse should visit the ward at the specified time every day to check whether the pipeline is unblocked or falling off. The drainage bag should be replaced in time every day to prevent infection. The color and shape of the drainage fluid should be monitored every day and reported to the doctor if there is any abnormality. (3) *Action Guidance*. The nurse should tell the patient to stay in bed for at least 48 hours after the operation. The patient should not try to get out of bed and move on the ground. After the patient was stable, he was asked to perform appropriate activities on the ground. (4) *Discharge Guidance.* The patient was informed to strictly control his diet after discharge, and he was provided dietary guidance to prevent indigestion caused by excessive food.

### 2.3. Main Instruments and Reagents

The main reagents and instruments in this study include adrenocorticotropic hormone (ACTH) kit (BYabscience, Nanjing of China), cortisol kit (Shanghai Jining Biotechnology Co., Ltd.), ether (Shandong Chu Xin Chemical Co., Ltd.), estradiol reference substance (Guangzhou Jiatu Technology Co., Ltd.), testosterone reference substance (Solarbio Life Science, Beijing of China), phosphate-buffered saline solution (Hubei Chengfeng Chemical Co., Ltd.), centrifuge (Beijing Haiyi Technology Co., Ltd.) , ultralow temperature refrigerator (Jinan Alaboo Instrument Equipment Co., Ltd.), radioimmunoassay counter (Hefei Zhongcheng Electromechanical Technology Development Co., Ltd.), constant temperature water bath (Jinan Tongxin Biological Technology Co., Ltd.), and electric oscillator (Shanghai Following Spectrum Electronic Technology Co., Ltd.).

### 2.4. Determination of Hormone Content

8 mL of peripheral venous blood was drawn from all patients on the second day after admission and on the 1^st^, 3^rd^, 6^th^, 15^th^, and 30^th^ day after surgery.

The CTH detection was performed as follows. 2 mL of serum was taken into a test tube containing 30 *μ*L of ethylenediaminetetraacetic acid disodium, shaken gently to mix well, centrifuged at 3000 rpm for 10 min to separate the serum, and then stored in a refrigerator at −80°C. 15–20 minutes before the start of the experiment, the sample was put in room temperature or ice water to remelt and centrifuged at 3000 rpm for 5 min to take the supernatant. 100 *μ*L was placed into the special test tube for radioimmunoassay. In addition, the phosphate buffered saline solution, ACTH standard product, serum to be tested, 125I-ACTH, and rabbit anti-ACTH antiserum were injected into the empty tube, standard product test tube, and serum sample tube, which were shaken gently to mix well and then placed in a water bath at 4°C for at least 15 hours. Then, after 500 *μ*L of rabbit anti-immune separation reagent was injected into each test tube, it was shaken to mix and incubated at room temperature for 15 min and centrifuged at 3000 rpm/centrifuge for 10 min to remove the supernatant. Finally, the radioactive substance count in each test tube was measured.

The cortisol detection was performed as follows. 10 minutes before the experiment, the kit and the sample to be tested were taken out of the refrigerator and cooled to room temperature. 100 *μ*L of sample was placed into the special radioimmunoassay tube. In addition, the phosphate buffered saline solution, ACTH standard product, serum to be tested, 125I-ACTH, and rabbit anti-ACTH antiserum were injected into the empty tube, standard product test tube, and serum sample tube, which were shaken gently to mix well and then placed in a water bath at 37°C for 50 hours. The subsequent operations were the same as the ACTH determination process.

The estradiol detection was performed as follows. 3-4 mL of serum was collected and placed in a 37°C water bath for 40 min and then centrifuged at 3000 rpm for 5 min to separate the plasma, which was injected into the test tube, sealed, and stored in a −76°C refrigerator. In the experiment, 200 *μ*L of standard substance and serum samples to be tested were injected into the test tubes, and 1 mL of phosphate buffered saline solution was injected into each tube, shaken gently until fully mixed, and then incubated at room temperature for 10 min. After 2.5 mL of distilled ether was added to each tube, it was quickly covered tightly to avoid volatilization, and then it was placed in an electric shaker and vigorously shaken for 2 min. After stratification was found, the ether was placed in the test tube in a refrigerator at −20°C for 35 min. The ether of the extracted hormone in the upper part of the liquid was injected into a brand new test tube, and all the liquid was evaporated with nitrogen in a 37°C water bath. After the test tube was taken out, 200 *μ*L of phosphate buffer saline solution was injected and incubated at room temperature for 10 min. Then, 200 *μ*L was aspirated for extraction and determination strictly according to the instructions.

The testosterone detection was performed with the same operations as the estradiol determination process.

### 2.5. CT Examination

All patients were informed to fast for 8 hours and to refrain from drinking for 6 hours before the examination and were required to take about 1500 mL of water 30 min before the examination to fill the upper gastrointestinal tract. The patient lied on his back on the examination table with his feet advanced, his arms raised and placed on both sides of his head, and the patient was asked not to move and keep his breathing steady. The Revolution CT Machine (GE Company, USA) was used to scan the patient's diaphragm from the top of the diaphragm to the lower edge of the liver, with the upper horizontal line under the xiphoid process and both sides at the midaxillary level. The scanning parameters were determined as follows: tube voltage was switched between 80 kVp and 140 kVp, tube current was 50 mA, arteriovenous phase was 480 mA, layer thickness was 4 mm, spacing was 5 mm, and pitch was 0.992 : 1.

All images were processed by GE adw4.6 work station to reconstruct the iodine/water-based substance map, and the iodine/water concentration of normal liver tissue, blood supply area, and necrotic area on the image were measured. Three experienced professional imaging physicians were invited to take the test three times, and the average value of the data was taken.

### 2.6. Recursive Residual Coding and Decoding Algorithm Based on Deep Learning

For an image with noise, it can be simply regarded as the aliasing of a clear image and noise, which can be expressed as follows:

(1) $$\begin{array}{c} I=A+N. \end{array}$$

In the above equation, *N* represented the noise, *A* represented the clear image, and *I* referred to the image with interference noise obtained in the image inspection. The noise in the image was generally Gaussian noise, including fluctuating noise, cosmic noise, thermal noise, and shot noise. The probability density function of its normal distribution was expressed as follows:

(2) $$\begin{array}{c} p\left(z\right)=\frac{1}{\sqrt{2\pi }\sigma }e^{-{\left(z-\bar{z}\right)}^{2}/2\sigma^{2}}. \end{array}$$

However, the noise in CT images generally appears as striped artifacts, which do not conform to the standard of normal distribution. Therefore, the usual means of removing Gaussian noise to remove the noise of CT images will generally not be too good, so it has to find a suitable method for denoising.

Convolutional neural network (CNN) is a neural network structure, which calculates input data through multilayer nonlinear mapping and outputs prediction results. The essence is a regression optimization calculation, which introduces a feedback layer into the traditional multilayer perception network structure to optimize the prediction results. However, the common CNN has a shortcoming; that is, when the depth of the neural network increases, the network performance will appear to be in a state of no change or even decline. The residual network is added with the jump connections to the network to avoid the disadvantage of gradient disappearance during backpropagation, thereby improving the performance of the network. The biggest difference between the residual network and the ordinary CNN is that the latter directly obtains the denoised image, while the residual network extracts the residual between the clear image and the noisy image with more concise method and relatively small calculation amount. The basic structure was shown in Figure 1.

The residual network is formed by providing a basic set of residual units, containing two stacked convolutional layers. It was assumed that *O*_*n*_ was the input of the n-th residual unit, *O*_*n*+1_ was the output result, *F*(*O*) represented the residual mapping of the convolutional layer, and *Q*_*n*_ referred to the weight of the *n*-th layer. Then, the entire relationship can be expressed as follows:

(3) $$\begin{array}{c} O_{n+1}=O_{n}+F\left(O_{n},\left\{Q_{n}\right\}\right). \end{array}$$

If the dimensionality of the image processed by the stacked convolutional layer cannot be consistent with the original image, then the dimensionality mapping convolutional layer was required in the jump connection. This convolution kernel can be represented by the *H*_*s*_, which was expressed as follows:

(4) $$\begin{array}{c} O_{n+1}=F\left(O_{n},\left\{Q_{n}\right\}\right)+H_{s}O_{n}. \end{array}$$

By analogy, from level 0 to level *n*, equation (3) can be summarized by *O*_*N*_=*O*_*o*_+∑_*i*=0_^*N*−1^*F*(*O*_*i*_, *H*_*i*_). Used together with jump connection, linear transformation can be used to connect the input and output layers at one time. When the depth of the network was equal, the operation difficulty of the residual network was the same as that of the ordinary network, and there was no need to learn other parameters, but the residual network can design the deeper network architecture.

When a common network was applied to denoise an image, there was no way to completely remove the noise in the image at one time. Therefore, based on the residual network, the content of the residual codec network was combined with the recursive network in this study to build a new network model, which was named as recursive residual encoder-decoder network (RRED-Net). It not only had the advantages of the residual network (easy to train) but also combined the advantages of the recursive network. It can repeat the denoising processing on the original input image, and it can also restore the details of the image to the greatest extent.

It was assumed that *M* ∈ *T*^*U*×*V*^ represented a general CT image and *N* ∈ *T*^*U*×*V*^ represented a normal dose CT image. Then, the process of image quality degradation can be expressed as follows:

(5) $$\begin{array}{c} M=\vartheta \left(N\right). \end{array}$$

In the equation above, *ϑ* represented the direct mapping from *N* to *M*.

The noise removal process of a general CT image can be regarded as an end-to-end mapping problem. When the image *M* was inputted, a mapping *g* satisfaction can be obtained after the training of the residual network, which was expressed as follows:

(6) $$\begin{array}{c} \arg\min{\left\|g\left(M\right)-N\right\|}_{2}^{2}. \end{array}$$

In the equation above, *g* was the approximation of *ϑ*^−1^ and *N* referred to the CT image of normal dose. In the residual network, *g*(*M*)=*G*(*M*)+*M*, and the residual mapping *G*(*M*) was obtained after network training, which was the residual between the general CT image *M* and the normal dose CT image *N*.

Then, in this overall architecture, the residual codec network in equation (6) can be repeatedly used to denoise the image. In each recursion, the initial image and the output result of the *y*-th recursion were regarded as the input of the next recursion, which can avoid the loss of information in the initial image during the recursive process, extract image features more completely, and retain detail. The recursive process of the residual network can be expressed as follows:

(7) J1=M,On=KRE  D−NetJn 1≤n<N,Jn+1=kinO,nM 1≤n<N.

In the equation above, *n* represented the total number of recursion, *M* represented the network input, RED-Net was the residual codec network built, *O*_*n*_ referred to the noise-free CT image obtained after the n-th recursion, and *k*_*in*_ represented the cascading reaction between the output result *O*_*n*_ of the n-th recursion and the initial general CT image *M*. *J*_*n*+1_ represented the input for the *n* + 1-th recursion. For the evaluation of the processed image quality, the peak signal-to-noise ratio (PSNR) and the structural similarity index (SSIM) were selected to judge the performance of the denoising algorithm used. The definition of PSNR was as follows:

(8) $$\begin{array}{c} \text{PSNR}=10\;\log_{10}\frac{D}{\sqrt{\left(1/UV\right)\sum {}_{i=0}^{u-1}\sum {}_{j=0}^{v-1}{\left[C\left(i,j\right)-E\left(i,j\right)\right]}^{2}}}. \end{array}$$

In the above equation, *C* represented an image without noise in *u* × *v*, *E* referred to an image processed by denoising, and *D* referred to the absolute value of the difference between the maximum and minimum pixel values of the image.

The definition of SSIM was as follows:

(9) $$\begin{array}{c} \text{SSIM}=\frac{\left(2\lambda_{p}\lambda_{\hat{p}}+z_{1}\right)\left(2\gamma_{p\hat{p}}+z_{2}\right)}{\left(\lambda_{p}^{2}+\lambda_{\hat{p}}^{2}+z_{1}\right)\left(\gamma_{p}^{2}+\gamma_{\hat{p}}^{2}+z_{2}\right)}. \end{array}$$

In the above equation, *λ*_*p*_ and $\lambda_{\hat{p}}$ represented the average value of the images *p* and $\hat{p}$, respectively; *z*_1_ and *z*_2_ were prescribed numbers; *γ*_*p*_ and $\gamma_{\hat{p}}$ referred to the variance between the images *p* and $\hat{p}$, respectively; and $\gamma_{p\hat{p}}$ referred to the covariance of the images *p* and $\hat{p}$.

### 2.7. Observation Index

After a period of nursing, the indexes were observed, including blood supply area, necrosis area, ACTH level, cortisol level, estradiol level, testosterone level, SAS score, and compliance as comparison and quality of life score detected by CT in the two groups.

### 2.8. Statistical Analysis

All experimental data were statistically analyzed by SPSS 24.0, measurement data were expressed as mean + standard deviation ($\bar{x}$ ± *s*), and the count data were used for statistical inference using *χ*^2^ test. The measurement data conforming to normal distribution was performed with the *t*-test. *P* < 0.05 was considered statistically significant difference.

## 3. Results

### 3.1. Comparison of General Information of the Two Groups of Patients

As shown in Table 1, there was no great difference between the control and experimental groups in terms of age, gender, tumor size, history of liver cirrhosis, length of surgery, and number of lesions, which were not statistically significant (*P* > 0.05).

### 3.2. Comparison on the Presence or Absence of Blood Supply to the Lesions between the Two Groups of Patients

The CT imaging technology based on intelligent algorithm was used to examine the lesions of the two groups of patients after the operation. The detection situation was shown in Figure 2. There were 95 lesions in the control group, including 86 blood supply areas, and nine necrotic areas were detected, so the necrosis rate was 9%. There were a total of 98 lesions in the experimental group, including 92 blood supply areas, and six necrotic areas were detected, so the necrosis rate was 6%. The FNR of the experimental group was lower than that of the control group, and the difference was statistically significant (*P* < 0.05).

### 3.3. Comparison of Neuroendocrine Hormone Levels between the Two Groups at Each Time Point

As shown in Figure 3, there was no obvious difference in the levels of neuroendocrine hormone (ACTH, cortisol, estradiol, and testosterone) between the two groups of patients before surgery, which was not statistically observable (*P* > 0.05). After the surgery, the levels of ACTH of the experimental group were not significantly different from those of the control group at T1, T2, and T5. The levels of ACTH at T3 and T4 were 41.25 ± 3.81 pg/mL and 19.55 ± 1.72 pg/mL, respectively, which were lower than those in the control group, which were 46.21 ± 3.97 pg/mL and 28.82 ± 2.16 pg/mL, respectively (*P* < 0.05). The cortisol levels of the experimental group were not dramatically different at T1 and T2 in contrast to the control group; at T3, T4, and T5, the levels of cortisol were 424.86 ± 16.82 nmol/L, 277.98 ± 14.36 nmol/L, and 241.53 ± 13.27 nmol/L, respectively, so all of which were lower than those in the control group, which were 452.42 ± 17.9 nmol/L, 309.83 ± 15.72 nmol/L, and 270.34 ± 13.02 nmol/L (*P* < 0.05). The estradiol levels of the experimental group were not remarkably different from those of the control group at T1 and T2, which were 53.48 ± 11.19 pg/mL, 41.64 ± 9.28 pg/mL, and 30.59 ± 8.16 pg/mL at T3, T4, and T5, respectively, so all were lower than those of the control group, which were 58.77 ± 11.52 pg/mL, 47.59 ± 9.31 pg/mL, and 39.78 ± 8.44 pg/mL, respectively (*P* < 0.05). The testosterone levels of the experimental group were not significantly different from those of the control group at T1 and T2, which were 2.18 ± 1.14 ng/mL, 1.78 ± 1.03 ng/mL, and 1.42 ± 0.69 ng/mL at T3, T4, and T5, respectively, so all were lower in contrast to the control group, which were 2.65 ± 1.07 ng/mL, 2.14 ± 0.98 ng/mL, and 1.92 ± 0.73 ng/mL, respectively (*P* < 0.05).

### 3.4. Comparison of SAS Scores of Patients in Each Group at Each Time Point

Self-Rating Anxiety Scale (SAS) is a standard for anxiety assessment and is a psychological scale used to measure the degree of anxiety and its changes. Patients whose anxiety scores were below 50 were determined as normal condition, patients whose scores were 50–60 points were determined as mild anxiety, patients whose scores were 61–70 points were considered as moderate anxiety, and patients whose scores were above 70 points were diagnosed as severe anxiety. As shown in Figure 4, there was no obvious difference in the SAS scores of the two groups of patients before surgery, which was not statistically remarkable (*P* > 0.05). After surgery, the SAS scores of the experimental group were not greatly different from those of the control group at T1 and T2, which were 40.24 ± 5.81 points, 36.55 ± 5.02 points, and 32.53 ± 4.8 points at T3, T4, and T5, respectively, and they were lower than those of the control group (46.11 ± 5.76 points, 40.42 ± 4.88 points, and 37.84 ± 4.79 points, respectively), showing statistically remarkable differences (*P* < 0.05).

### 3.5. Comparison of Compliance Behavior between the Two Groups of Patients

As illustrated in Figure 5, the numbers of patients in the experimental group in terms of no smoking and drinking, taking medication on time, diet control, and self-monitoring were 24, 27, 23, and 21, respectively, which were all higher than those in the control groups (20 cases, 24 cases, 18 cases, and 17 cases, respectively), so the differences were statistically obvious (*P* < 0.05).

### 3.6. Comparison on Quality of Life Scores between Two Groups of Patients before and after Surgery

Figure 6 illustrates the comparison on quality of life scores between two groups of patients before and after surgery.  Figure 7(a) suggests that there was no visible difference in the quality of life scores between the two groups of patients before surgery, showing no statistical difference (*P* > 0.05). After the surgery, the physical function, self-cognition, emotional function, and social function scores of patients in the experimental group were 62.59 ± 6.82 points, 69.26 ± 8.14 points, 73.89 ± 6.35 points, and 66.88 ± 7.04 points, respectively; and those in the control group were 50.68 ± 6.72 points, 61.33 ± 7.29 points, 65.38 ± 6.21 points, and 60.17 ± 6.26 points, respectively (Figure 7(b)). Thus, the scores of patients for physical function, self-cognition, emotional function, and social function in the experimental group were much higher in contrast to the control group, and the differences were statistically great (*P* < 0.05).

### 3.7. Comparison of CT Images before and after Surgery Processed by Intelligent Algorithm

There was a 62-year-old male patient in the experimental group who complained of pain and discomfort in his right upper abdomen for more than 3 months and was admitted to the hospital with progressive aggravation. Preoperative CT examination showed that there was a mass in the liver and the intrahepatic bile ducts were dilated. The image display was unclear, and there was interference noise inside, which affected the reading of the film. After the image was processed with the intelligent algorithm based on the residual network, most of the dorsal side of the lesion was ablated, and there were fewer residual lesions. The image was clearly displayed and there was no unwanted noise (Figure 7). After undergoing humanized nursing for one month after the surgery, the patient gained 4 kg in weight.

## 4. Discussion

Neuroendocrine hormone is one of the important hormones to maintain the stability of human environment. It participates in many physiological processes such as growth, development, and biochemical metabolism [16]. Neuroendocrine hormones can regulate the transcription of a variety of genes and protein synthesis and promote the growth of hormone dependent tumors [17]. The liver is the target organ of a variety of hormones and the main site for biological transformation and storage of hormones. The imbalance of hormone level in the body can often cause changes in cell biological effects [18], which leads to the occurrence of tumors, and tumor tissues can also secrete “ectopic hormones.” This change of hormone level can cause hypothalamic pituitary axis imbalance, thus further affecting the hormone level in the body [19]. In this study, 60 patients with primary liver cancer after operation were randomly divided into routine nursing control group (30 cases) and humanized nursing experimental group (30 cases). Through a period of nursing, the two groups of patients were evaluated by CT image based on intelligent algorithm and hormone content in blood. The results showed that the levels of ACTH, cortisol, estradiol, and testosterone in the control group were higher than those in the experimental group (*P* < 0.05). The main reason may be that, under routine nursing, the recovery speed of damaged liver function was slower than humanized nursing, and the excess neuroendocrine hormones in the body could not be effectively inactivated, resulting in the accumulation of hormones in the body. In this research, a recursive shallow residual codec network model was constructed to remove artifacts and noise in CT images, and a new algorithm was proposed. On the one hand, by reducing the number of layers and convolution cores in the residual codec network, the complexity of the network was reduced, and the recursive idea was used to obtain high-quality images. On the other hand, in order to avoid the loss of details caused by convolution and better reconstruct the image, the original input image was cascaded to the next input at each recursion. The experimental results showed that recursive artifact removal was an effective method, which could not only reduce the complexity of the network but also improve the performance of the network, so that the denoising results could preserve the image details and have a clearer structure.

There are many postoperative complications of liver cancer. Failure to strengthen nursing will affect the prognosis of patients, thus affecting the quality of life of patients. The results of this study showed that the quality of life score of patients with whole process humanized nursing was significantly higher than that of patients with routine nursing (*P* < 0.05). The activity guidance helps the patients not to get out of bed prematurely, which leads to bleeding at the surgical site, strengthens the management of the drainage bag, replaces the drainage bag every day, prevents the occurrence of infection, and optimizes the prognosis, so as to improve the physical function and social function of the patients. Psychological nursing was carried out for patients to improve their self-awareness and strengthen their self-confidence, so as to improve their self-awareness and emotional function score. Yan's study showed that the blood oxygen saturation of jaundiced newborns with humanized nursing intervention was better than that of children with routine nursing intervention [20]. The results of this study were consistent with it. The survival rate of patients with liver cancer within 5 years after operation was low, and they were easy to relapse after operation. Patients were worried about their survival status and have symptoms such as anxiety and depression. Improving patients' negative emotion is very meaningful in the follow-up treatment of cancer surgery. The results of this study showed that the scores of anxiety and depression after hepatectomy with the whole process humanized nursing intervention were lower than those under routine nursing, indicating that the whole process humanized nursing can improve the negative emotions of patients. Nurses give psychological guidance to patients with whole process humanized nursing intervention to help them strengthen self-awareness and improve self-confidence. At the same time, it also gives psychological comfort to patients' families and urges their families to give patients more psychological support. Previous studies had shown that the anxiety and depression scores of patients in cardiovascular surgery intensive care unit under humanized nursing were significantly lower than those in routine nursing [21]. The results of this study were consistent with those of previous studies. Humanized nursing process can improve postoperative patients' compliance, optimize quality of life, relieve patients' anxiety, depression, and other adverse emotions, and play a positive role in patients' neuroendocrine hormones and prognosis.

## 5. Conclusion

In this study, 60 postoperative patients with primary liver cancer were randomly divided into the same amount of routine nursing group and humanized nursing group. Through a period of nursing, the hormone content was determined and evaluated by using CT images based on intelligent algorithm. The results showed that the experimental group was better than the control group in local necrosis rate, neuroendocrine hormone level at some time points, SAS score at some time points, postoperative compliance, and quality of life score, and the difference was statistically significant (*P* < 0.05). In the future, the sample size will be expanded to conduct more in-depth research in this direction.

## Figures and Tables

**Figure 1:** The basic structure of residual network.

**Figure 2:** Comparison on the presence or absence of blood supply to the lesions between the two groups of patients. Note. :indicates that the detection of lesions in the experimental group showed a statistically significant difference compared with the control group (*P* < 0.05).

**Figure 3:** Comparison of neuroendocrine hormone levels between the two groups at each time point. (a) The comparison of preoperative overall levels; (b–e) the comparisons of postoperative ACTH levels, cortisol levels, estradiol levels, and testosterone levels, respectively. ^*∗*^indicates that the hormone level of the experimental group was statistically significant compared with that in the control group (*P* < 0.05).

**Figure 4:** Comparison of SAS scores before and after operation between the two groups. (a, b) The comparison on SAS score at each time point before and after the surgery, respectively. ^*∗*^suggests that the SAS score in the experimental group showed statistical difference in contrast to that in the control group (*P* < 0.05).

**Figure 5:** Comparison of compliance behavior between the two groups of patients. ^*∗*^indicates that the compliance of patients in experimental group was statistically different from that in the control group (*P* < 0.05).

**Figure 6:** Comparison on quality of life scores between two groups of patients before and after surgery. (a, b) The comparison on quality of life scores of two groups of patients before and after the surgery, respectively. ^*∗*^indicates that the quality of life score of patients in experimental group was statistically different from that in the control group (*P* < 0.05).

**Figure 7:** Comparison of CT images before and after surgery. (a, b) Preoperative CT images; (c, d) postoperative CT images processed by intelligent algorithms.

**Table 1:** Comparison of general information of the two groups of patients.

	Control group	Experimental group	*P*
Age (years)	48.38 ± 2.74	47.86 ± 2.85	0.768
Male (people)	24	22	0.744
Tumor size (cm)	6.87 ± 1.22	6.54 ± 1.31	0.639
Cirrhosis (weeks)	21	22	0.692
Operation time (h)	2.92 ± 0.81	2.94 ± 0.76	0.727
Focuses	95	98	0.684

## Data Availability

The data used to support the findings of this study are available from the corresponding author upon request.
